RETRACTED

# Thiazole-valine peptidomimetic (TTT-28) antagonizes multidrug resistance *in vitro* and *in vivo* by selectively inhibiting the efflux activity of ABCB1

**DOI:** 10.1038/srep42106

**Published:** 2017-02-09

**Authors:** Yi-Jun Wang, Bhargav A. Patel, Nagaraju Anreddy, Yun-Kai Zhang, Guan-Nan Zhang, Saeed Alqahtani, Satyakam Singh, Suneet Shukla, Amal Kaddoumi, Suresh V. Ambudkar, Tanaji T. Talele, Zhe-Sheng Chen

**Affiliations:** 1 Department of Pharmaceutical Sciences, College of Pharmacy and Health Sciences, St. John’s University, Queens, NY 11439, USA; 2 Department of Basic Pharmaceutical Sciences, School of Pharmacy, The University of Louisiana at Monroe, Monroe, LA 71201, USA; 3 Laboratory of Cell Biology, Center for Cancer Research, National Cancer Institute, National Institutes of Health, Bethesda, Maryland, MD 20892, USA

## Abstract

Multidrug resistance (MDR) attenuates the chemotherapy efficacy and increases the probability of cancer recurrence. The accelerated drug efflux mediated by ATP-binding cassette (ABC) transporters is one of the major MDR mechanisms. This study investigated if TTT-28, a newly synthesized thiazole-valine peptidomimetic, could reverse ABCB1-mediated MDR *in vitro* and *in vivo*. TTT-28 reversed the ABCB1-mediated MDR and increased the accumulation of [^3^H]-paclitaxel in ABCB1 overexpressing cells by selectively blocking the efflux function of ABCB1, but not interfering with the expression level and localization of ABCB1. Animal study revealed that TTT-28 enhanced the intratumoral concentration of paclitaxel and promoted apoptosis, thereby potently inhibiting the growth of ABCB1 overexpressing tumors. But TTT-28 did not induce the toxicity (cardiotoxicity/myelosuppression) of paclitaxel in mice. In this study, we synthesized and evaluated a novel selective inhibitor of ABCB1 (TTT-28) with high efficacy and low toxicity. The identification and characterization of this new thiazole-valine peptidomimetic will facilitate design and synthesis of a new generation of ABCB1 inhibitors, leading to further research on multidrug resistance and combination chemotherapy. Furthermore, the strategy that co-administer MDR-ABCB1 inhibitor to overcome the resistance of one FDA approved, widely used chemotherapeutic paclitaxel, may be promising direction for the field of adjuvant chemotherapy.

Cancer is a rapidly progressing disease. The American Cancer Society reported over 14.1 million new cancer cases and 7.6 million cancer deaths worldwide in 2014. Lung cancer ranks as the leading cause of cancer deaths, followed by breast and colorectal cancer. Cancer is constitutive of around two hundred invasive, heterogeneous diseases that originate in certain organs (e.g., lung, breast, colorectum, prostate) rather than a single disease^1^. Chemotherapy is one of the treatment choices apart from surgery and radiation. Chemotherapeutic drugs can conquer cancer via targeting the rapidly-dividing cancer cells and interfering with the cell proliferation. During chemotherapy, a unique phenomenon called multidrug resistance (MDR) emerges, in which cancer cells develop resistance to drugs with different chemical structures and mechanisms of action^2^. Development of MDR has been attributed to the failure of chemotherapy in over 90% of patients with metastatic cancer. It can attenuate the chemotherapy efficacy and raise the possibility of cancer recurrence^3^. The mechanisms of MDR are very sophisticated and consist of 1) increased metabolism of anticancer drug to its inactive metabolite; 2) alteration in the drug target, where the drug cannot bind to the target to produce the desired effect; 3) enhanced DNA damage repair leading to suppressed apoptosis; 4) alteration in the cell-cycle check points; 5) decreased drug uptake into the cells or increased drug efflux out of cells thereby diminishing the amount of drug in the intracellular region^4^,^5^. The ATP-binding cassette (ABC) transporter is primarily responsible for the drug efflux. It consists of 48 members that are classified into 7 subfamilies starting from ABCA through G, based on structural and sequence similarities^2^. Among them, ABCB1, ABCG2, ABCC1 and ABCC10 are the major inducers of MDR in cancer cells^6^,^7^. The main function of these transporters is to protect the normal cells against toxic substances. However, cancer cells overexpress ABC transporters and exploit them to export anticancer drugs out of cells, thereby protecting themselves. ABC transporters force drugs out of cells against the concentration gradient using ATP (adenosine triphosphate). In the presence of a substrate drug, the ATP hydrolysis occurs and leads to conformational changes in the transporter. During the open conformation, it exports drugs out of cells. Soon the second molecule of ATP returns the transporter to its original high-affinity conformation and it is ready to transport drug again^8^.

RETRACTED

ABCB1 (P-gp/MDR1) is an apical membrane transporter that is ubiquitously expressed in kidney, intestine, placenta, liver, adrenal glands and blood-brain barrier (BBB)^3^,^9^. Overexpression of ABCB1 has been found to trigger MDR and exhibit resistance to diverse substrate anticancer drugs, like anthracyclines, vinca alkaloids, taxanes, epipodophyllotoxins, TKIs (tyrosine kinase inhibitors)^6^,^9^. Several reports revealed the close connection between ABCB1 overexpression and assorted cancers, such as advanced gastrointestinal stromal tumor (GIST), non-small cell lung cancer (NSCLC), fallopian tube, ovarian and thyroid cancer^10^,^11^,^12^,^13^,^14^. Successful chemotherapy can only be accomplished on condition that optimal pharmacokinetics, tumor penetration and intracellular concentrations are conserved inside cancer cells. Hence it is essential to develop modulators of ABC transporters that can increase the intracellular concentration of anticancer drugs. The clinical significance of ABCB1 transporter antagonism has been studied as a potential therapeutic strategy.

In our previous study, 21 novel compounds were synthesized by peptide coupling at the corresponding carboxyl and amino termini of (*S*)-valine-based bis-thiazole and monothiazole derivatives with diverse chemical scaffolds^15^. Importantly, this structure-activity relationship (SAR) study resulted in identification of TTT-28 (compound **28** in Singh *et al*.^15^) bearing a trimethoxybenzoyl moiety and a 2-amino benzophenone moiety at the amino and carboxyl termini of the monothiazole zwitter-ion (Fig. 1A). The calcein-AM efflux and MTT assays demonstrated that TTT-28 was the most effective ABCB1 inhibitor among the synthesized compounds. Docking analysis indicated interactions of TTT-28 within site-1 in the drug-binding pocket of homology-modeled human ABCB1^15^. Since above findings showed that TTT-28 potently reversed ABCB1-mediated MDR *in vitro*, we were interested to find answers to clinically relevant questions related to the reversal effect of TTT-28: (1) What is the mechanism of action inside the cancer cells? (2) Does TTT-28 affect the expression level or translocation of ABCB1? (3) How does TTT-28 affect the function of ABCB1? (4) Can this *in vitro* activity be translated to *in vivo* models (efficacy vs. toxicity)? (5) What are the pharmacodynamics and pharmacokinetics parameters of TTT-28? Through obtaining answers to these questions, this study would provide a perspective on MDR-reversal mechanism of TTT-28 in cancer cells.

## Results

### Effect of TTT-28 on sensitization to ABCB1 substrates in cell lines overexpressing ABCB1

To select a non-toxic drug concentration for TTT-28, cytotoxicity assays were performed on the cell lines (Supplementary Fig. 1). Based on these results, 5 μM and 10 μM were chosen, because more than 85% of the cells survived at 10 μM. To determine whether TTT-28 can reverse ABCB1-mediated MDR, MTT assays were performed using human colon cancer cell line SW620 and doxorubicin-resistant subline SW620/Ad300. SW620/Ad300 cell line exhibited 631.9−, 268.5− and 168.6-fold resistance to paclitaxel, doxorubicin, vincristine (ABCB1 substrates), respectively, as compared to SW620 cell line. TTT-28 at 10 μM dramatically decreased the resistance fold of paclitaxel, doxorubicin, vincristine down to 1.9, 2.8, 1.7, respectively in SW620/Ad300 cells (Table 1). Importantly, TTT-28 (10 μM) almost completely reversed ABCB1-mediated MDR in SW620/Ad300 cells. The reversal effects of TTT-28 at both 5 μM and 10 μM were stronger than that of verapamil (positive control inhibitor of ABCB1) at 10 μM. No significant changes were observed in the IC_50_ for SW620 and SW620/Ad300 when TTT-28 or verapamil was combined with cisplatin (not a substrate of ABCB1).

RETRACTED

MDR can be induced by various factors^16^. To exclude other factors and focus on the sole factor ABCB1, we used HEK293/pcDNA3.1 and ABCB1-transfected HEK/ABCB1 cells. The similar phenomenon was observed in this pair of cell lines. TTT-28 produced a concentration-dependent reduction in ABCB1-mediated resistance to paclitaxel, doxorubicin and vincristine in HEK/ABCB1 cells (Table 1). These results suggested that TTT-28 potently resensitized ABCB1 overexpressing both drug selected and transfected cells to ABCB1 substrate anticancer drugs. Supplementary Table 1 showed that TTT-28 was more cytotoxic to colon cancer cells than human normal colon fibroblast cells CCD-18Co. SW620 and SW620/Ad300 cells were more susceptible to combination treatment than CCD-18Co, indicating that combination treatment not only possessed improved anticancer efficacy, but also favorable anticancer selectivity (Supplementary Table 2).

### Effect of TTT-28 on reversal of drug resistance in cell lines overexpressing ABCG2, ABCC1 and ABCC10

To determine the effect of TTT-28 on ABCG2, we used HEK293/pcDNA3.1 and ABCG2 transfected wild-type ABCG2-482-R2 cells. Fumitremorgin C (FTC) is a specific, selective, and potent inhibitor at micromolar concentrations of ABCG2 transporter^17^. TTT-28 did not significantly alter the IC_50_ values of HEK293/pcDNA3.1 and ABCG2-482-R2 cells to topotecan. However, FTC significantly decreased the resistance of ABCG2-482-R2 to topotecan (Supplementary Table 3). Hence TTT-28 did not reverse ABCG2-mediated MDR. Next, we used HEK/ABCC1 and HEK/ABCC10 cells to demonstrate that TTT-28 had no reversal effect on the ABCC1- or ABCC10-mediated MDR. PAK-104P is a potent inhibitor of ABCC1/MRP1^18^. Cepharanthine is a potent reversal agent for ABCC10/MRP7-mediated multidrug resistance^19^.

### TTT-28 does not change the expression level and localization of ABCB1

To investigate that the reversal of ABCB1-mediated MDR by TTT-28 was not caused by downregulation of ABCB1, we treated cells with TTT-28 (10 μM) for 0, 24, 48 and 72 h. No obvious alteration in the expression level of ABCB1 was observed in drug-selected SW620/Ad300 and transfected HEK/ABCB1 cells (Fig. 1B).

RETRACTED

If ABCB1 was translocated from the membrane to the cytosolic region, one would expect diminished expression of membrane ABCB1. To test this potential mechanism, the immunofluorescence assay was conducted to investigate if the location of ABCB1 was changed after the incubation of SW620/Ad300 cells with TTT-28. Shown in Fig. 1C, TTT-28 did not trigger the internalization of cell surface ABCB1. These important findings disclosed that the MDR reversal mechanism of TTT-28 was not induced by the alteration in the expression and localization of ABCB1, but may result from blocking the efflux function of ABCB1.

### Effect of TTT-28 on cellular accumulation of [^3^H]-paclitaxel

To study the effect of TTT-28 on ABCB1 substrates, accumulation assay was conducted to measure intracellular drug concentration. Intracellular concentration of [^3^H]-paclitaxel was significantly increased from 0.05 to 1.31 pmol/10^6^ cells in SW620/Ad300 after TTT-28 (10 μM) treatment (Fig. 2A). Consistent with MTT results, the intracellular accumulation of 5 μM and 10 μM TTT-28 groups was significantly higher than that of 10 μM verapamil group.

### TTT-28 inhibits the efflux activity of ABCB1 transporter

To confirm whether increase in the intracellular accumulation was induced by inhibiting the efflux of [^3^H]-paclitaxel, the drug efflux assay was performed with reversal agent at different time points (0, 30, 60, 120 min). The remaining intracellular amount of [^3^H]-paclitaxel in SW620/Ad300 was significantly lower compared to that of SW620 cells resulting from the active efflux by ABCB1. Intracellular remaining [^3^H]-paclitaxel was greatly increased from 20.4% to 57.9% in SW620/Ad300 after 10 μM TTT-28 treatment for 120 min (Fig. 2B).

### Effect of TTT-28 on the ATPase activity of ABCB1

To assess the effect of TTT-28 on the ATPase activity of ABCB1, we measured ABCB1-mediated ATP hydrolysis in the presence of TTT-28 at various concentrations (0–40 μM). TTT-28 stimulated the ATPase activity of ABCB1 in a concentration dependent fashion, with a maximal stimulation of 3.38-fold of the basal activity. The inset in Fig. 2C demonstrated that the concentration of TTT-28 required to obtain 50% stimulation was 0.652 ± 0.053 μM. In addition, photoaffinity labeling of ABCB1 with [^125^I]-IAAP (Iodoarylazidoprazosin) assay in our previous study indicated TTT-28 binds at the drug-binding pocket located in the transmembrane domains of human ABCB1^15^. Hence TTT-28 interacts at the drug-substrate-binding site and affects the ATPase activity of ABCB1.

### TTT-28 significantly potentiates the anticancer activity of paclitaxel in an ABCB1 overexpressing tumor xenograft model

To investigate the efficacy of TTT-28, paclitaxel, and combination of paclitaxel with TTT-28, tumor xenograft mouse models were used. Mice bearing SW620 and SW620/Ad300 tumors were administered with 30 mg/kg TTT-28, 15 mg/kg paclitaxel, or combination. Figure 3A and B showed that tumor volumes of SW620 tumors after the 18-day treatment of vehicle, TTT-28, paclitaxel, and combination of paclitaxel and TTT-28 were 2096.1 mm^3^, 1954.8 mm^3^, 604.3 mm^3^ and 416.7 mm^3^, respectively (Fig. 3A and B). The tumor weights of SW620 tumors after the 18-day treatment of vehicle, TTT-28, paclitaxel, and combination were 2.82 g, 2.73 g, 0.75 g and 0.50 g (Fig. 3C). Combination treatment exhibited more potent inhibitory effect than paclitaxel alone on the growth of SW620 tumors.

RETRACTED

Figure 4A and B showed that the tumor volumes of SW620/Ad300 tumors after the 18-day treatment of vehicle, TTT-28, paclitaxel, and combination were 2194.2 mm^3^, 2113.4 mm^3^, 1280.8 mm^3^ and 526.2 mm^3^. The tumor weights of SW620/Ad300 tumors after the 18-day treatment of vehicle, TTT-28, paclitaxel, combination were 3.02 g, 2.89 g, 1.53 g and 0.60 g (Fig. 4C). These data indicated that TTT-28 greatly potentiated the inhibitory effect of paclitaxel on the growth of SW620/Ad300 tumors.

### TTT-28 significantly raises paclitaxel concentration in tumors but not in plasma of the ABCB1 overexpressing tumor xenograft model

To investigate the effect of TTT-28 on paclitaxel pharmacokinetics, we measured the plasma and intratumoral concentrations of paclitaxel in animals pretreated with paclitaxel, combination of paclitaxel with TTT-28. No significant difference in the SW620 intratumoral concentration of paclitaxel was observed between paclitaxel group (416.5 ng/mL) and combination group (476.0 ng/mL). Interestingly, TTT-28 greatly enhanced the SW620/Ad300 intratumoral concentration of paclitaxel (215.5 ng/ml) as compared to paclitaxel alone group (46.8 ng/ml, *P* < 0.01) at 240 min after administration (Fig. 5A). This is consistent with the results of [^3^H]-Paclitaxel accumulation assay. However, TTT-28 did not significantly affect the plasma concentration of paclitaxel (Fig. 5B). These results indicated that TTT-28 induced increment in the efficacy of paclitaxel in SW620/Ad300 tumors is primarily due to its inhibitory effect on the efflux function of ABCB1, leading to higher intratumoral accumulation of paclitaxel.

To study the effect of paclitaxel on TTT-28 pharmacokinetics, we measured the plasma and intratumoral concentrations of TTT-28 in mice. In SW620 and SW620/Ad300 tumors, no significant variation in the intratumoral concentration of TTT-28 was found between TTT-28 group and combination group (Fig. 5C). Mean concentration of TTT-28 in SW620/Ad300 tumors was significantly higher than that in SW620 tumors. Similar to tariquidar, TTT-28 might be a unique ABCB1 inhibitor. Distinct from other ABCB1 substrates, binding of TTT-28 at a site within the drug-binding pocket would enable it to stabilize both TMDs (transmembrane domains, enhanced corrector activity) and bring the two wings and NBDs (nucleotide-binding domains) together into a closed conformation that would result in stimulation of ATPase activity but no efflux activity (inhibitor)^20^. Stabilization of the first TMD by TTT-28 could be an important mechanism that explains the stronger reversal effect and significant increase in the accumulation of TTT-28 in SW620/Ad300 tumors as compared to SW620 tumors. In addition, paclitaxel moderately increased the plasma concentration of TTT-28 (Fig. 5D).

RETRACTED

### Evaluation of TTT-28 toxicity in tumor xenograft mice model

No apparent weight loss was observed among four treatment groups (Fig. 5E). Thus administration of TTT-28, paclitaxel, combination of TTT-28 and paclitaxel did not produce any visible toxicity or phenotypic changes in mice. Since myelosuppression (neutropenia and thrombocytopenia) are the common adverse effects of paclitaxel, we conducted blood smear test to investigate the number of white blood cells (WBC) and platelets in mice. It has been reported that the normal range of WBC and platelets in mice are 1.32 × 10^9^~8.38 × 10^9^ WBC/L and 0.7 × 10^11^~12.0 × 10^11^ platelets/L^21^. The mean numbers of WBC and platelets in paclitaxel alone and combination groups were significantly lower than that in vehicle group (Fig. 5F and G). However, mean numbers of WBC and platelets in four treatment groups were all in the normal range, disclosing that TTT-28 and combination treatment would not induce neutropenia or thrombocytopenia in mice.

It is well known that one of the most dangerous side effects of paclitaxel is cardiomyopathy, leading to congestive heart failure^22^. Cardiac troponin-I (cTnI) is often used as a marker to indicate the damage of cardiac muscle^23^. Figure 6A showed the cTnI levels of TTT-28 group were similar to those of vehicle group, indicating that TTT-28 had no cardiotoxicity. The cTnI levels of combination group were slightly lower than those of paclitaxel group, which had moderate cardiotoxicity.

### *Ex vivo* immunohistochemistry (IHC) analysis of SW620 and SW620/Ad300 tumor tissues

IHC analysis was performed to further evaluate the *in vivo* antitumor activity. Shown in Fig. 6B, paclitaxel and combination group displayed obvious nuclear condensation and fragmentation in the H&E (hematoxylin and eosin) images. Paclitaxel and combination groups upregulated the expression levels of ABCB1 in SW620 tumors after the 18-day treatment. The active caspase-3 and cleaved PARP-1 staining indicated that paclitaxel and combination groups induced the higher level of apoptosis in SW620 tumors, as compared to vehicle and TTT-28 group (Supplementary Fig. 3A,C and E). Figure 6C showed that combination group displayed higher level of nuclear condensation and fragmentation than paclitaxel group. Paclitaxel and combination groups did not upregulate the expression levels of ABCB1 in SW620/Ad300 tumors after 18-day treatment. The active caspase-3 and cleaved PARP-1 staining indicated that combination group induced the highest level of apoptosis in SW620/Ad300 tumors, as compared to other three groups (Supplementary Fig. 3B,D and F). Thus these IHC analyses are supportive of the prominent anticancer efficacy of the combination treatment.

RETRACTED

## Discussion

As primary contributor of MDR, ABCB1 constitutes a defense program to pump out chemotherapeutic agents from cells. It is necessary to develop ABCB1 modulators that can circumvent MDR via inhibiting the efflux activity of ABCB1. This approach will increase the efficacy of antineoplastic drugs and cure rate of chemotherapy. Multiple methods (random and focused screening, systemic chemical modifications, combinatorial chemistry) have been utilized to develop the first three generations of ABCB1 inhibitors, but they failed in clinical trials. Many of them were inhibitors of CYP3A4 and enhanced the plasma concentration of co-administered anticancer drugs which deteriorated toxicity. Some of these drugs were non-specific and inhibited other ABC transporters that resulted in more severe side effects of anticancer drugs^24^. The clinical failures were also because of low bioavailability at tumor microenvironment^25^, nonspecific inhibition of ABCB1 expressed in all tissues including BBB, and improper selection of the patient population^26^. To overcome these issues, new strategies to facilitate the development of fourth generation ABCB1 inhibitors possessing high ABCB1 selectivity and efficacy are urgently required. One useful strategy is to attach distinct chemical fragments that are usually found in ABCB1 inhibitors to a new chemotype like thiazole amino acid. The selection of the fragments was based on the chemical moieties that are always seen in reported preclinical and clinical candidates such as tariquidar, elacridar, LY402913, reserpine, XRR9051, saracatinib, galloyl-based inhibitors and benzophenone derivatives^15^.

RETRACTED

In this study, we established an ABCB1 overexpressing tumor xenograft mouse model to demonstrate that TTT-28 can inhibit the efflux activity of ABCB1 transporter, thereby significantly increasing the intratumoral concentration of paclitaxel and potentiating the antineoplastic activity of paclitaxel. Firstly, *in vitro* studies assays proved that TTT-28 (10 μM) can nearly completely reverse ABCB1-mediated MDR in both drug selected SW620/Ad300 cells and transfected HEK/ABCB1 cells. Secondly, TTT-28 was tested to show no reversal effect on the ABCG2-, ABCC1-, ABCC10-mediated MDR. In other words, the reversal effect of TTT-28 is potent and specific to ABCB1. TTT-28 raised the accumulation of [^3^H]-paclitaxel in ABCB1 overexpressing cells by blocking the efflux function of ABCB1, without interfering with the expression level and localization of ABCB1. TTT-28 stimulated the basal ATP hydrolysis of ABCB1 in a concentration-dependent fashion.

To translate these valuable findings into *in vivo* models, we began with the tumor xenograft mouse model. To determine the vehicle to deliver TTT-28 *in vivo*, we measured the aqueous solubility of TTT-28 at pH 7.4 to be 0.5 mg/mL. PEG300 was used as a solubilizing agent for the oral delivery of TTT-28. The procedure for aqueous solubility study is described in the Supplementary experimental procedures section. Paclitaxel and combination treatment can shrink SW620 tumors by 3.76 times and 5.64 times as compared to vehicle control group. Paclitaxel and combination treatment can inhibit the growth of SW620/Ad300 tumors by 1.97 times and 5.03 times. The only 1.97 times inhibition of paclitaxel on the SW620/Ad300 tumors is much smaller than the 3.76 times shrinkage of SW620 tumors by paclitaxel, indicating that the ABCB1 overexpressing SW620/Ad300 tumors are resistant to paclitaxel treatment. The 5.03 times inhibition of combination therapy is significantly higher than the 1.97 times inhibition of paclitaxel on SW620/Ad300 tumors. These *in vivo* results show high clinical values for the co-administration of TTT-28 and ABCB1 substrate antineoplastic drugs in ABCB1-mediated MDR cancer patients. Pharmacokinetic study demonstrated that TTT-28 greatly enhanced the concentration of paclitaxel inside the SW620/Ad300 tumors.

TTT-28 did not induce the toxicity (cardiotoxicity/myelosuppression) of paclitaxel. IHC analysis of tumor sections demonstrated that combination group promoted apoptosis in SW620/Ad300 tumors. Since there is a high probability of P-gp inhibitors being CYP3A4 inhibitors too, we determined whether TTT-28 has such an inhibitory effect. We found that TTT-28 inhibits CYP3A4 with an IC_50_ of 8.23 ± 0.37 μM.

RETRACTED

In conclusion, TTT-28 is a novel selective inhibitor of ABCB1 with high efficacy and low toxicity. These findings reveal high clinical value for the co-administration of TTT-28 and ABCB1 substrate chemotherapeutic drugs in cancer patients that overexpress ABCB1 and stimulate further research on circumventing multidrug resistance and ABC transporter.

## Materials and Methods

### Chemicals and equipment

[^3^H]-paclitaxel (23 Ci/mmol) was purchased from Moravek Biochemicals, Inc. (Brea, CA). Paclitaxel, doxorubicin, vincristine, cisplatin, topotecan, verapamil, Triton X-100, paraformaldehyde, DMSO, MTT were obtained from Sigma Chemical Co. (St. Louis, MO). The monoclonal antibody C219 (against ABCB1), sc-47778 (against β-Actin) and the secondary horseradish peroxidase-labeled rabbit anti-mouse IgG were purchased from Santa Cruz Biotechnology, Inc. (Dallas, TX). The Alexa flour 488-conjugated goat anti-mouse IgG was purchased from Molecular Probes (Eugene, OR). WBC Diluting Fluid and Platelet Diluent were purchased from Eng Scientific Inc. (Clifton, NJ). High sensitivity mouse cardiac troponin-I ELISA KIT was purchased from Life Diagnostics, Inc. (West Chester, PA). SAView^@^ (mouse/rabbit-HRP, DAB) IHC kit was obtained from Enzo Life Sciences, Inc. (Farmingdale, NY). OPSYS microplate reader was purchased from Dynex Technologies (Chantilly, VA).

### Cell lines and cell culture

The SW620/Ad300 cell line overexpressing ABCB1, was established by a step-wise exposure of SW620, the parental human colon cancer cell line, to increasing concentration of doxorubicin up to 300 μg/L. HEK293/pcDNA3.1, wild-type ABCG2-482-R2 was established by selection with G418 after transfecting HEK293 with empty pcDNA3.1 vector and the pcDNA3.1 vector containing the full-length ABCG2, coding arginine at amino acid position 482. HEK/ABCB1, HEK/ABCC1 and HEK/ABCC10 cells were generated by transfecting the HEK293 cells with ABCB1, ABCC1 and ABCC10 expression vector, respectively. Transfected cells were selected in DMEM containing 2 mg/ml G418^27^. The human normal colon fibroblast cell line CCD-18Co was cultured at 37 °C, 5% CO2, with EMEM containing 10% FBS and 1% penicillin/streptomycin.

### Cell viability assay

The sensitivity of cells to anticancer drugs was measured as previously described using the MTT colorimetric assay^28^.

### Western blot analysis

60 μg protein cell lysates were resolved using 8–12% sodium dodecyl sulfate polyacrylamide gel electrophoresis (SDS-PAGE) and transferred onto polyvinylidene fluoride (PVDF) membranes through electrophoresis. ABCB1 was determined from C219, and β-Actin was used as internal loading control as previously mentioned in Zhang *et al*.^29^.

RETRACTED

### Immunofluorescence assay

Cells (1 × 10^4^ cells per well) were seeded into 96-well plate. After TTT-28 treatment, cells were fixed with 4% paraformaldehyde for 15 min at room temperature (RT) and then rinsed with PBS. Then cells were kept in 1% Triton X-100 for 10 min at 4 °C. Non-specific reactions were blocked with BSA (2 mg/ml) for 1 h at 37 °C. The monoclonal antibody against ABCB1 was applied overnight, followed by an Alexa flour 488-conjugated goat anti-mouse IgG for 1 h. Propidium iodide was used to counterstain the nuclei. Images were taken with Nikon TE2000 inverted microscope (Nikon Instruments Inc. Melville, NY)^30^.

### [^3^H]-Paclitaxel accumulation and efflux assay

The accumulation of [^3^H]-paclitaxel in SW620 and SW620/Ad300 cells was measured in the absence or presence of TTT-28 or verapamil at 5 μM and 10 μM. The drug accumulation and efflux assay were performed as described previously^31^.

### ABCB1 ATPase assay

The vanadate-sensitive ATPase activity of ABCB1 in crude membranes of High-five insect cells, in the presence of concentrations of TTT-28 ranging from 0 to 40 μM, was measured as previously described^32^.

### Animal preclinical antitumor efficacy trial design

The SW620 and SW620/Ad300 models were designed with some modification of the tumor xenograft model previously established by Chen and colleagues^33^. There were four treatment groups. Group 1 animals received the vehicle A (polyethylene glycol 300/N-methyl pyrrolidone/saline, 22.5%/2.5%/75%) orally every 3rd days, 1 hour prior to intraperitoneal administration of vehicle B (ethanol/Cremophor ELP/saline, 12.5%/12.5%/75%). Group 2 animals received 30 mg/kg TTT-28 orally (prepared in vehicle A) administered every 3rd day, 1 hour prior to intraperitoneal administration of vehicle B. Group 3 animals received the vehicle A orally every 3rd day, 1 hour prior to 15 mg/kg intraperitoneal paclitaxel administration. Group 4 animals received combination of the TTT-28, administered every 3rd day orally, 1 hour prior to intraperitoneal paclitaxel administration. Eight mice were used for each group. The tumor sizes were measured using calipers and body weights were recorded^34^. The body weight of the animals was monitored every third day to adjust the drug dosage and to determine treatment-related toxicities as well as disease progression. The two perpendicular diameters of tumors were recorded every third day and the tumor volume was estimated^35^. Later all mice were euthanized using carbon dioxide, tumor tissues were excised and stored at −80 °C. All mice were maintained at the St. John’s University Animal Facility. The IACUC at St. John’s University approved this project, and the research was conducted in compliance with the Animal Welfare Act and other federal statutes.

RETRACTED

### Tumor and plasma collection

Mice bearing SW620 and SW620/Ad300 tumors were divided into three groups: (i) TTT-28; (ii) paclitaxel; (iii) TTT-28 + paclitaxel. After treatment, animals were anesthetized and blood was obtained using supraorbital puncture and placed in heparinized tubes and plasma was harvested at 10, 30, 60, 120, or 240 min after paclitaxel administration in both groups.

### Quantification of TTT-28 and paclitaxel

The quantification of TTT-28 in plasma and tumors was conducted using an isocratic Shimadzu LC-20AB HPLC equipped with a Shimadzu SIL-20A HT autosampler and LC-20AB pump connected to a Dgu-20A3 degasser (Shimadzu, OR). A reverse-phase, Phenomenex Luna C18 column (250 × 4.6 mm i.d., 5 μm; Phenomenex, CA) with an ODS guard column (4 mm × 3 mm; Phenomenex, CA), was used. The injection volume was 20 μl, and the mobile phase used for the separation of TTT-28 in plasma and tissue homogenate samples consisted of acetonitrile and water (90:10, v/v) delivered at a flow rate of 1.0 ml/min. For TTT-28 detection, the Shimadzu UV SPD-20A (Shimadzu, OR) detector set was at 210 nm. Data acquisition and analysis was achieved using LC Solution software version 1.22 SP1 (Shimadzu, OR). All samples were analyzed in duplicate. Under these chromatographic conditions, the total run time was 10 min with a retention time of 5.6 min for TTT-28. Standard curves for TTT-28 in plasma and tissue homogenates were prepared in the ranges of 10–10,000 ng/ml. The preparation and storage of samples and quantification of paclitaxel in tumor and plasma were performed as previously described^36^.

### Blood cell counting

The platelets and WBCs in mice were counted as described previously^33^.

### Mouse cardiac troponin-I ELISA assay

The plasma with heparin was prepared after blood collection and stored at 4 °C. The desired number of coated wells in the holder was secured and 100 μl of cTnl HRP Conjugate was dispensed into each well. Then 100 μl of standards and diluted samples were dispensed into appropriate wells and incubated on an orbital shaker (150 rpm) at RT for 60 min. Later, the incubation mixture was removed by flicking the plate contents into a waste container. The microtiter wells were washed and emptied 6 times with 1x wash solution. After washing, the wells were struck sharply onto absorbent paper to remove all residual droplets. 100 μl of TMB reagent were dispensed into each well and incubated at RT for 20 min on an orbital shaker at ~150 rpm. The reaction was stopped by adding 100 μl Stop Solution to each well. The mixture was gently mixed and the absorbance was read at 450 nm with a microtiter well reader^33^.

RETRACTED

### Immunohistochemistry (IHC) analysis

The IHC analysis of SW620 and SW620/Ad300 tumors was performed as previously described^33^.

### Statistical analysis

All experiments were repeated at least three times, each done in triplicate. The statistical significance between two groups was determined with Student’s t-test, whereas the comparisons of multiple groups was carried out by one-way ANOVA, followed by Bonferroni’s post-test using Microsoft Excel software. A probability value of *P < 0.05 was considered to be significant.

## Additional Information

**How to cite this article**: Wang, Y.-J. *et al*. Thiazole-valine peptidomimetic (TTT-28) antagonizes multidrug resistance *in vitro* and *in vivo* by selectively inhibiting the efflux activity of ABCB1. *Sci. Rep.* **7**, 42106; doi: 10.1038/srep42106 (2017).

**Publisher's note:** Springer Nature remains neutral with regard to jurisdictional claims in published maps and institutional affiliations.

## Supplementary Material

Supplementary Information

## Figures and Tables

**Figure 1:** (**A**) Chemical structure of TTT-28. (**B**) Western blot analysis showing the effect of TTT-28 at 10 μM on the expression levels of ABCB1 in both SW620/Ad300 and HEK/ABCB1 cells for 0, 24, 48 and 72 h. Equal amounts (60 μg) of cell lysates were loaded into each well and subjected to Western blot analysis as described in “Materials and Methods” section. Representative result is shown here and similar results were obtained in two other independent trials. The full-length blots are shown in Supplementary Fig. 5. (**C**) The immunofluorescence assays showing the effect of TTT-28 at 10 μM on the subcellular localization of ABCB1 in SW620/Ad300 cells for 72 h.

**Figure 2:** (**A**) The accumulation of [^3^H]-paclitaxel was measured after the cells (parental SW620 and ABCB1 overexpressing SW620/Ad300 drug selected cell lines) were pre-incubated with or without TTT-28 or verapamil for 2 h at 37 °C and then incubated with 0.01 mM [^3^H]-paclitaxel for another 2 h at 37 °C. Columns are the mean of triplicate determinations; error bars represent SD. *P < 0.05 versus control group (blue column, SW620/Ad300), ^#^*P* < 0.05 versus group of 5 μM verapamil (yellow column, SW620/Ad300); one-way ANOVA with Bonferroni post-test. (**B**) The effect of TTT-28 or verapamil on the efflux of [^3^H]-paclitaxel from SW620 and SW620/Ad300 cells. Cells were pre-treated with or without TTT-28 or verapamil at 10 μM for 2 h at 37 °C and further incubated with 0.01 mM [^3^H]-paclitaxel at 37 °C for 2 h. Cells were then incubated in the fresh medium with or without the reversal agents for different time periods at 37 °C. Cells were then collected and the intracellular levels of [^3^H]-paclitaxel were determined by scintillation counting. A time course versus percentage of intracellular [^3^H]-paclitaxel remaining (%) was plotted (0, 30, 60, 120 min). Lines are the mean of triplicate determinations; error bars represent SD. *P < 0.05 versus control group (blue dash line); one-way ANOVA with Bonferroni post-test. TTT-28 is tested compound as ABCB1 inhibitor. Verapamil is a positive control of ABCB1 inhibitor. (**C**) Crude membranes (100 μg protein/ml) from High-five cells expressing ABCB1 were incubated with increasing concentrations of TTT-28 (0–40 μM), in the presence and absence of sodium orthovanadate (Vi) (0.3 mM), in ATPase assay buffer as described in “Materials and Methods” section. The graph shows that ATPase activity was plotted with SD as a function of concentration of TTT-28. The inset shows stimulation of ATP hydrolysis at lower (0–10 μM) concentration of TTT-28.

RETRACTED

**Figure 3:** The effect of TTT-28 and paclitaxel on the growth of SW620 tumors in nude athymic mice. (**A**) The images of excised SW620 tumors implanted subcutaneously in athymic NCR nude mice (n = 8) that were treated with vehicle, TTT-28, paclitaxel and the combination of TTT-28 and paclitaxel, at the end of the 18-day treatment period. (**B**) The changes in tumor volume over time following the implantation. Data points represent the mean tumor volume for each treatment group (n = 8). Error bars, SEM. *P < 0.05 versus the vehicle group; ^#^*P* < 0.05 versus the paclitaxel group; one-way ANOVA with Bonferroni post-test. (**C**) The mean weight (n = 8) of the excised SW620 tumors from the mice treated with vehicle, TTT-28, paclitaxel and the combination of TTT-28 and paclitaxel, at the end of the 18-day treatment period. Error bars, SEM. *P < 0.05 versus the vehicle group; ^#^*P* < 0.05 versus the paclitaxel group; one-way ANOVA with Bonferroni post-test.

**Figure 4:** The effect of TTT-28 and paclitaxel on the growth of SW620/Ad300 tumors in nude athymic mice. (**A**) The images of excised SW620/Ad300 tumors implanted subcutaneously in athymic NCR nude mice (n = 8) that were treated with vehicle, TTT-28, paclitaxel and the combination of TTT-28 and paclitaxel, at the end of the 18-day treatment period. (**B**) The changes in tumor volume over time following the implantation. Data points represent the mean tumor volume for each treatment group (n = 8). Error bars, SEM. *P < 0.05 versus the vehicle group; ^#^*P* < 0.05 versus the paclitaxel group; one-way ANOVA with Bonferroni post-test. (**C**) The mean weight (n = 8) of the excised SW620/Ad300 tumors from the mice treated with vehicle, TTT-28, paclitaxel and the combination of TTT-28 and paclitaxel, at the end of the 18-day treatment period. Error bars, SEM. *P < 0.05 versus the vehicle group; ^#^*P* < 0.05 versus the paclitaxel group; one-way ANOVA with Bonferroni post-test.

RETRACTED

**Figure 5:** The pharmacokinetic characteristics of TTT-28 and paclitaxel in the nude athymic mice. (**A**) Intratumoral paclitaxel concentrations in SW620 (n = 8) and SW620/Ad300 tumors (n = 8) after 240 min following administration of paclitaxel alone or the combination of TTT-28 and paclitaxel (n = 8). Columns and error bars represent mean ± SEM. *P < 0.05 versus the paclitaxel SW620 group; ^#^*P* < 0.05 versus the paclitaxel SW620/Ad300 group; one-way ANOVA with Bonferroni post-test. (**B**) Plasma paclitaxel concentrations in nude athymic mice at 10, 30, 60, 120, 240 min following administration of paclitaxel alone or the combination of TTT-28 and paclitaxel (n = 8). (**C**) Intratumoral TTT-28 concentrations in SW620 (n = 8) and SW620/Ad300 tumors (n = 8) after 240 min following administration of TTT-28 alone or the combination of TTT-28 and paclitaxel (n = 8). Columns and error bars represent mean ± SEM. *P < 0.05 versus the TTT-28 SW620 group; ^#^*P* < 0.05 versus the TTT-28 SW620/Ad300 group; one-way ANOVA with Bonferroni post-test. (**D**) Plasma TTT-28 concentrations in nude athymic mice at 10, 30, 60, 120, 240 min following administration of TTT-28 alone or the combination of TTT-28 and paclitaxel (n = 8). *P < 0.05 versus the TTT-28 group; Student’s t-test. The effect of TTT-28 and paclitaxel on the body weight, white blood cells and platelets in nude athymic mice. (**E**) The changes in mean body weight of mice (n = 8) before and after the treatment. NS, not statistically significant (P > 0.05). (**F**) The changes in mean white blood cells in nude mice (n = 8) at the end of the 18-day treatment period. (**G**) The changes in mean platelets in nude mice (n = 8) at the end of the 18-day treatment period. *P < 0.05 versus the vehicle group; one-way ANOVA with Bonferroni post-test.

**Figure 6:** *Ex vivo* immunohistochemistry (IHC) analysis of SW620 and SW620/Ad300 tumor sections and cardiotoxicity of TTT-28. (**A**) The changes in mean levels of cardiac troponin I in nude mice (n = 8) at the end of the 18-day treatment period. *P < 0.05 versus the vehicle group; ^#^*P* < 0.05 versus the paclitaxel group; one-way ANOVA with Bonferroni post-test. (**B**) SW620 and SW620/Ad300 tumor sections (**C**). In H&E staining, nuclei are stained blue, and extracellular matrix and cytoplasm are stained red. In ABCB1, Caspase-3 and PARP staining, nuclei are stained blue, and ABCB1, Caspase-3 and PARP are stained brown.

RETRACTED

**Table 1:** The reversal effect of TTT-28 and verapamil on the cytotoxicity of paclitaxel, doxorubicin, vincristine and cisplatin to SW620 and SW620/Ad300, HEK293/pcDNA3.1 and HEK/ABCB1 cell lines.

Treatment	SW620		SW620/Ad300		HEK293/pcDNA3.1		HEK/ABCB1	
	IC_50_ ± SD^a^ (μM)	FR^b^	IC_50_ ± SD (μM)	FR	IC_50_ ± SD (μM)	FR	IC_50_ ± SD (μM)	FR
Paclitaxel	0.007 ± 0.001	[1.0]	4.423 ± 0.218	[631.9]	0.049 ± 0.002	[1.0]	4.481 ± 0.234	[91.4]
+TTT-28 (5 μM)	0.007 ± 0.001	[1.0]	0.024 ± 0.002*	[3.4]	0.048 ± 0.003	[1.0]	0.135 ± 0.018*	[2.8]
+TTT-28 (10 μM)	0.007 ± 0.002	[1.0]	0.013 ± 0.002*	[1.9]	0.048 ± 0.002	[1.0]	0.085 ± 0.003*	[1.7]
+Verapamil (10 μM)	0.007 ± 0.001	[1.0]	0.027 ± 0.003*	[3.9]	0.048 ± 0.003	[1.0]	0.155 ± 0.021*	[3.2]
Doxorubicin	0.061 ± 0.003	[1.0]	16.378 ± 0.955	[268.5]	0.058 ± 0.002	[1.0]	4.076 ± 0.171	[70.3]
+TTT-28 (5 μM)	0.059 ± 0.004	[1.0]	0.324 ± 0.023*	[5.3]	0.057 ± 0.003	[1.0]	0.323 ± 0.017*	[5.6]
+TTT-28 (10 μM)	0.058 ± 0.004	[1.0]	0.171 ± 0.012*	[2.8]	0.057 ± 0.003	[1.0]	0.135 ± 0.031*	[2.3]
+Verapamil (10 μM)	0.059 ± 0.005	[1.0]	0.377 ± 0.019*	[6.2]	0.058 ± 0.003	[1.0]	0.354 ± 0.022*	[6.1]
Vincristine	0.025 ± 0.002	[1.0]	4.216 ± 0.289	[168.6]	0.028 ± 0.002	[1.0]	2.597 ± 0.254	[92.8]
+TTT-28 (5 μM)	0.025 ± 0.001	[1.0]	0.071 ± 0.005*	[2.8]	0.027 ± 0.003	[1.0]	0.079 ± 0.015*	[2.8]
+TTT-28 (10 μM)	0.025 ± 0.002	[1.0]	0.043 ± 0.005*	[1.7]	0.028 ± 0.003	[1.0]	0.051 ± 0.003*	[1.8]
+Verapamil (10 μM)	0.025 ± 0.003	[1.0]	0.076 ± 0.004*	[3.0]	0.027 ± 0.003	[1.0]	0.093 ± 0.006*	[3.3]
Cisplatin	1.234 ± 0.083	[1.0]	1.248 ± 0.177	[1.0]	1.372 ± 0.174	[1.0]	1.268 ± 0.147	[0.9]
+TTT-28 (5 μM)	1.280 ± 0.092	[1.0]	1.278 ± 0.114	[1.0]	1.347 ± 0.239	[1.0]	1.293 ± 0.152	[0.9]
+TTT-28 (10 μM)	1.272 ± 0.089	[1.0]	1.275 ± 0.142	[1.0]	1.376 ± 0.199	[1.0]	1.287 ± 0.108	[0.9]
+Verapamil (10 μM)	1.273 ± 0.148	[1.0]	1.285 ± 0.093	[1.0]	1.330 ± 0.237	[1.0]	1.337 ± 0.158	[1.0]

^a^IC_50_: concentration that inhibited cell survival by 50% (means ± SD).

^b^FR: fold-resistance represents IC_50_ value for paclitaxel, doxorubicin, vincristine, and cisplatin of SW620 and SW620/Ad300, HEK293/pcDNA3.1 and HEK/ABCB1 cells in the absence or presence of TTT-28 and verapamil was divided by IC_50_ value for paclitaxel, doxorubicin, vincristine, and cisplatin in parental SW620 or HEK293/pcDNA3.1 cells. Values in table are determined from at least three independent experiments performed in triplicate. Verapamil was used as a positive control of ABCB1 inhibitor. ^*^Indicates significantly different from IC_50_ of SW620/Ad300 or HEK/ABCB1 without reversal drug (*P < 0.05); one-way ANOVA with Bonferroni post-test.
